# A Modified Reptile Search Algorithm for Numerical Optimization Problems

**DOI:** 10.1155/2022/9752003

**Published:** 2022-10-10

**Authors:** Qihang Yuan, Yongde Zhang, Xuesong Dai, Shu Zhang

**Affiliations:** ^1^Key Laboratory of Advanced Manufacturing and Intelligent Technology, Ministry of Education, Harbin University of Science and Technology, Harbin 150080, China; ^2^Foshan Baikang Robot Technology Co., Ltd, Nanhai, Foshan, Guangdong 528225, China

## Abstract

The reptile search algorithm (RSA) is a swarm-based metaheuristic algorithm inspired by the encirclement and hunt mechanisms of crocodiles. Compared with other algorithms, RSA is competitive but still suffers from low population diversity, unbalanced exploitation and exploration, and the tendency to fall into local optima. To overcome these shortcomings, a modified variant of RSA, named MRSA, is proposed in this paper. First, an adaptive chaotic reverse learning strategy is employed to enhance the population diversity. Second, an elite alternative pooling strategy is proposed to balance exploitation and exploration. Finally, a shifted distribution estimation strategy is used to correct the evolutionary direction and improve the algorithm performance. Subsequently, the superiority of MRSA is verified using 23 benchmark functions, IEEE CEC2017 benchmark functions, and robot path planning problems. The Friedman test, the Wilcoxon signed-rank test, and simulation results show that the proposed MRSA outperforms other comparative algorithms in terms of convergence accuracy, convergence speed, and stability.

## 1. Introduction

The rapid advancement of technology has generated a large number of optimization problems that require solving. These optimization problems arise in various fields, such as finance, chemicals, electronics, machinery, and materials. Real-world optimization problems are often mixed with various unknown factors and have very complex solution spaces. These problems frequently have substantial computational efforts, complex nonlinear constraints, and large numbers of variables and constraints [1–6]. Traditional optimization methods have difficulty solving these nonproductivity discontinuity problems effectively because they cannot strike a balance between accuracy and time cost [7]. Metaheuristic optimization algorithms have demonstrated better performance in balancing the solution quality and time cost [8]. Due to a simple structure and no requirement for a problem to be continuously derivable, metaheuristic optimization algorithms have been widely used to solve complex optimization problems in natural and engineering fields [9–13].

In recent decades, metaheuristic algorithms have made great progress in memetic computing manner, balance of exploitation and exploration, self-adaption of hyperparameters, population structure evolution, and theoretical analysis of the search dynamics [14]. Memetic computing manner improves algorithm performance through metaheuristic algorithms incorporated with local search operator. Charin et al. used particle swarm optimization (PSO) combined with levy flight optimization (LFO) to track the maximum power point of a photovoltaic system [15]. Yu et al. showed that the combination of chaotic local search (CLS) and brain storm optimization (BSO) can significantly improve the performance of BSO [16]. How to balance the exploration and exploitation of the algorithm to improve the performance is a research hotspot of the metaheuristic algorithms. Many researchers use various operators or change the algorithm parameters to balance [17]. Cai et al. proposed an alternate search pattern strategy to balance the exploration and exploitation of BSO [18]. In the optimization process, the search performance of some metaheuristic algorithms is greatly affected by adjustable parameters such as crossover rate, mutation rate, and population size. In order to solve the problem of parameter value control at different stages in the optimization process, adaptive parameter control has been extensively studied by researchers [19]. Lei et al. proposed a variant of gravitational search algorithm (GSA) with a self-adaptive gravitational constant called ALGSA, which greatly improved the search performance of GSA [20]. Population structure evolution has great influence on the search performance of the metaheuristic algorithms. Zhong et al. proposed a variant to improve the performance of differential evolution (DE) algorithm called EHDE by incorporating elite elements into the hierarchical population structure [21]. Inspired by the two-layered structure GSA, Wang et al. proposed a four-layered GSA variant with stronger search capability called MLGSA [22]. In addition to the above factors, theoretical analysis of the search dynamics has recently attracted a great deal of attention from researchers [23].

In general, metaheuristic optimization algorithms can be classified into three categories [24]: evolutionary-based algorithms, physical-based algorithms, and swarm-based algorithms.

Evolutionary-based algorithms are inspired by the laws of natural evolution. Genetic algorithms are a typical example and their proposal was inspired by Darwinian evolutionary theory [25]. Genetic algorithms provide solutions through the concept of crossover and mutation of species in nature. In addition, other evolutionary-based algorithms have been proposed, including DE [26], evolutionary programming [27], and evolutionary strategies [28]. The second category is physics-based algorithms, which originate from natural physics laws. Simulated annealing [29] and GSA [30] are two common physics-based algorithms. They utilize the laws of thermodynamics and gravity for optimization. In addition, researchers have proposed other physics-based algorithms. Wei et al. proposed a nuclear reaction optimizer using the phenomenon of atomic nuclear reactions [31]. Inspired by the sine and cosine laws of mathematics, Mirjalili proposed the sine cosine algorithm [32]. Eskandar et al. proposed a water cycle algorithm based on the natural water cycle phenomena [33]. The third category is swarm-based algorithms, which build optimization models by emulating the social behavior of animal groups. PSO [34] and the ant colony algorithm [35] are two of the most common swarm-based algorithms. They provide solutions by sharing information about all individuals in the optimization process. Others include the grey wolf optimizer (GWO) [36], the whale optimization algorithm (WOA) [37], the butterfly optimization algorithm (BOA) [38], the firefly algorithm (FA) [39], the artificial bee colony (ABC) algorithm [40], the reptile search algorithm (RSA) [41], the Harris hawks optimizer (HHO) [42], the equilibrium optimizer (EO) [43], the tunicate swarm algorithm (TSA) [44], the salp swarm algorithm (SSA) [45], the Tasmanian devil optimization (TDO) [46], the arithmetic optimization algorithm (AOA) [47], and the pathfinder algorithm (PFA) [48].

The reptile search algorithm (RSA) is a novel swarm-based algorithm proposed by Abualigah. RSA is inspired by the encircling mechanism, hunting mechanism, and social behavior of crocodiles [41]. RSA has good performance but also has disadvantages such as diminished population diversity and unbalanced exploitation and exploration capabilities. To improve the performance of RSA and enhance the search capability, this paper proposes a modified variant of RSA, named MRSA. To improve the population diversity, an adaptive chaotic reverse learning strategy is proposed to optimize from the initialization and in each iteration update. To balance exploitation and exploration, an elite alternative pool strategy was developed. A shifted distribution estimation strategy was used to modify all the individuals and guide the evolutionary direction. To fully validate the performance of MRSA, 23 benchmark functions, IEEE CEC2017 benchmark functions, and robot path planning problems are used for testing. The superiority of the proposed algorithm is demonstrated by a convergence analysis, stability analysis, and statistical tests.

The rest of this paper is organized as follows.  Section 2 provides a review of the basic RSA. The proposed MRSA is described in detail in Section 3. In Section 4, the effectiveness of the proposed improved strategy and the superiority of the modified algorithm are verified using classical test functions, IEEE CEC2017 benchmark functions, and robot path planning problems. Finally, Section 5 provides the conclusion and discusses future work.

## 2. Reptile Search Algorithm

In this section, the basic procedures of RSA are presented. RSA is a swarm-based metaheuristic algorithm inspired by the enveloping mechanism, hunting mechanism, and social behavior of crocodiles.

### 2.1. Initialization Phase

RSA is similar to other metaheuristics in that the initial solution is generated randomly in the solution space. The initialization formula is as follows:

(1) $$\begin{array}{c} X_{i}^{1}=LB+rand\cdot \left(UB-LB\right)\text{,} \end{array}$$

where *X*_*i*_^1^ is the *i*^th^ initial individual and *LB* and *UB* are the upper and lower boundaries of the search space, respectively.

### 2.2. Encircling Phase (Exploration)

Crocodiles perform high and sprawl walks during the global search phase. In RSA, the search strategy is determined by the number of current iterations. When *t* ≤ 0.25*T*, RSA performs a high walk. When *t* ≤ 0.5*T* and *t* > 0.25*T*, the RSA performs a sprawl walk. The specific mathematical models of the mechanism are described as follows:

(2) $$\begin{array}{c} X_{i}^{t+1}=\left\{\begin{array}{c} X_{best}^{t}-\eta_{i}\times \beta -R_{i}^{t}\times rand,t\leq \frac{T}{4},\\ X_{best}^{t}\times X_{ran\;d}^{t}\times ES\times rand,t\leq \frac{T}{2}\;and\;t>\frac{T}{4}, \end{array}\right. \end{array}$$

(3) $$\begin{array}{c} \eta_{i}=X_{best}^{t}\times P_{i}\text{,} \end{array}$$

(4) $$\begin{array}{c} R_{i}=\frac{X_{best}^{t}-X_{i}^{t}}{X_{best}^{t}+\varepsilon }\text{,} \end{array}$$

(5) $$\begin{array}{c} ES=2\times r_{1}\times \left(1-\frac{1}{T}\right)\text{,} \end{array}$$

(6) $$\begin{array}{c} P_{i}=\alpha +\frac{X_{i}^{t}-M\left(X_{i}^{t}\right)}{X_{best}^{t}\times \left(UB-LB\right)+\varepsilon }\text{,} \end{array}$$

where *X*_best_^*t*^ is the current best solution, *t* is the current number of iterations, *T* is the maximum number of iterations, *β* is a constant taking the value of 0.1 to control the speed of exploration, *X*_ran d_^*t*^ is a randomly chosen individual, *ES* is a random value decreasing in the interval [−2, 2], *ε* is a minimal value to ensure that the denominator is not equal to 0, *r*_1_ is a random number in the interval [−1, 1], *α* is a constant taking the value of 0.1, and rand is a random number with values from 0 to 1.

### 2.3. Hunting Phase (Exploitation)

In RSA, crocodiles use two strategies for foraging: hunting coordination and cooperation. When *t* < 0.75*T* and *t* ≥ 0.5*T*, the RSA performs hunting coordination. When *t* < *T* and *t* ≥ 0.75*T*, a hunting cooperation strategy is employed by the RSA. The formula for position updating in the hunting phase is as follows:

(7) $$\begin{array}{c} X_{i}^{t+1}=\left\{\begin{array}{c} X_{best}^{t}\times P_{i}\times rand,t\leq \frac{3T}{4}\;and\;t>\frac{T}{2},\\ X_{best}^{t}-\eta_{i}\times \varepsilon -R_{i}^{t}\times rand,t\leq T\;and\;t>\frac{3T}{4}. \end{array}\right. \end{array}$$

RSA generates the initial population randomly in the search space first and then chooses different search strategies depending on the number of iterations. The pseudocode for the RSA is shown in Algorithm 1.

## 3. The Proposed RSA Variant

To enhance the performance of the basic RSA, three improvement strategies are proposed in this paper. An adaptive chaotic reverse learning strategy is first introduced to enhance the population diversity of RSA using the characteristics of chaotic mapping and reverse learning. Second, an elite alternative pooling strategy is used to balance the development and exploration of RSA. In addition, a distribution estimation strategy is used to modify the evolutionary direction. By sampling the dominant population information, the population direction is better guided, thus improving the algorithm's convergence efficiency. The three improvement strategies are described in detail in the following.

### 3.1. Adaptive Chaotic Reverse Learning Strategy

One of the shortcomings of the metaheuristic algorithm is that the diversity of the algorithmic population continues to diminish as the optimization proceeds. To enhance the diversity of the algorithms, the researchers employ different approaches. The reverse learning strategy is a new technique that is widely used to improve population diversity. The reason for the popularity of reverse learning is that extensive literature shows that the probability of a reverse solution approximating the global optimum is approximately fifty percent higher than the current original solution, and reverse learning strategies have been used to improve other algorithms with success [49–51]. The mathematical model of the reverse learning strategy is described as follows:

(8) $$\begin{array}{c} X_{i}^{o}=LB+UB-X_{i}^{t}\text{,} \end{array}$$

where *X*_*i*_^*o*^ is the inverse solution corresponding to *X*_*i*_^*t*^. The population diversity is related to the distribution of individuals in the search space. The more uniform the distribution of the individuals, the better the diversity. Chaotic mappings are characterized by random selection and ergodicity, which can help RSA generate new solutions and avoid premature convergence, and chaotic mappings have been successfully used to improve other algorithms [52]. Therefore, this paper combines a reverse learning strategy with chaotic mappings, called the chaotic reverse learning strategy, and it is given as follows:

(9) $$\begin{array}{c} X_{i}^{co}=LB+UB-\lambda_{i}X_{i}^{t}\text{,} \end{array}$$

where *X*_*i*_^*co*^ denotes the solution generated by the chaotic reverse learning mechanism corresponding to the *i*^th^ individual in the population. *λ*_*i*_ is the corresponding chaotic mapping value. There are ten common chaotic mappings, with the formulas and numerical distributions shown in Table 1.

For swarm-based algorithms, the quality of the initial population has a significant impact on the algorithm's performance. Therefore, the initial population is first generated using COBL to improve the population quality and to increase the algorithm's convergence accuracy. Second, during each iteration, the corresponding reverse population is generated using COBL and evaluated separately to retain the dominant individuals in the next generation.

In addition, as the algorithm proceeds, there will be many useless searches using the chaotic inverse learning strategy for all the individuals, which increases the computational cost and is not conducive to the convergence of the algorithm, so this paper proposes using the linear decreasing population strategy. As the iteration proceeds, the number of individuals using the chaotic inverse learning strategy is gradually reduced, and the specific mathematical formula is as follows:

(10) $$\begin{array}{c} Pop=round\left(\frac{\left(pop_{\min}-pop_{\max}\right)\cdot t}{T}+pop_{\max}\right)\text{,} \end{array}$$

where *Pop* denotes the number of populations using the chaotic backward learning strategy and *pop*_max_ and *pop*_min_ denote the maximum number and minimum number of populations, respectively.

### 3.2. Elite Alternative Pool Strategy

RSA performs position updates by following the best individual. This facilitates a faster convergence of the algorithm but diminishes population diversity and tends to trap local optimums. To maintain a balance between the exploitation and exploration of the algorithm, an elite alternative pooling strategy is proposed in this section. We place the current best three individuals into a pool as shown in the following equation:

(11) $$\begin{array}{c} X_{eap}=\left\{X_{eap1},X_{eap2},X_{eap3}\right\}\text{,} \end{array}$$

where *X*_*eap*1_, *X*_*eap*2_, and *X*_*eap*3_ are the three best individuals in the population thus far. The food source is chosen randomly from these three individuals each time. By using the elite alternative pooling strategy, the position of the food source changes from the best individual to one of the best three individuals. This goes some way to avoiding the premature convergence of the algorithm due to the best individual falling into a local optimum. To better balance the development and exploration of the algorithm, we also put the globally optimal individuals into the elite alternative pool to ensure that each individual has the opportunity to move closer to the optimal individual and ensure the convergence efficiency of the algorithm. Thus, the final mathematical model of the elite alternative pooling strategy is described as follows:

(12) $$\begin{array}{c} X_{eap}=\left\{X_{eap1},X_{eap2},X_{eap3},X_{best}\right\}\text{.} \end{array}$$

### 3.3. Shifted Distribution Estimation Strategy

RSA searches by following the optimal individuals, ignoring valid information from other individuals. To make full use of the position information of the dominant population, some scholars use a distribution estimation strategy for implementation [53, 54]. This strategy uses the current dominant population to calculate a probability distribution model, generates a new offspring population based on the sampling of the probability distribution model, and eventually obtains the optimal solution through continuous iteration. In addition to using the dominant population, this paper considers a modification of it by introducing information about the optimal individual and its own position and proposes a shifted distribution estimation strategy. The mathematical model is as follows:

(13) $$\begin{array}{c} \begin{array}{c} X_{i}^{t+1}=mean+y,y∼N\left(0,Cov\right)\text{,}\\ mean=\frac{\left(X_{best}^{t}+X_{mean}^{t}+X_{i}^{t}\right)}{3}\text{,}\\ Cov\left(i\right)=\frac{1}{NP/2}\overset{NP/2}{\underset{i=1}{\sum }}\left(X_{i}^{t+1}-X_{mean}^{t}\right)\times {\left(X_{i}^{t}-X_{mean}^{t}\right)}^{T}\text{,}\\ X_{mean}^{t}=\overset{NP/2}{\underset{i=1}{\sum }}\omega_{i}\times X_{i}^{t}\text{,}\\ \omega_{i}=\frac{\ln\;\left(0.5NP+0.5\right)-\ln\left(i\right)}{\overset{\begin{array}{c} NP/2 \end{array}}{\underset{i=1}{\sum }}\left.\left(\ln\left(0.5\right.NP+0.5\right)-\ln\;i\right)} \end{array} \end{array}$$

where *X*_mean_^*t*^ denotes the weighted position of the dominant population and *ω*_*i*_ denotes the weight coefficient in the dominant population in descending order of fitness values. **Cov** is the weighted covariance matrix of the dominant populations. The flow chart of MRSA is shown in Figure 1 and its pseudocode is in Algorithm 2.

### 3.4. Time Complexity

The time complexity determines the operating efficiency of the algorithm. In RSA, the computational complexity of the initialization process is *O*(*N*), where *N* is the population size. The computational complexity of the update process is *O*(*T* × *N*)+*O*(*T* × *N* × *D*), where *D* is the problem's dimensionality and *T* is the maximum number of iterations, so the computational complexity of RSA is *O*(*N* × (*T* × *D*+*T*+1)).

The computational complexity of MRSA is determined by six main factors (initialization process, solution update, number of fitness evaluations, chaotic reverse learning strategy, elite alternative pooling strategy, and shifted distribution estimation strategy). The computational complexity of the MRSA initialization process is *O*(*N*). The computational complexity of the update process is *O*(*T* × *N*)+*O*(2 × *T* × *N* × *D*). Therefore, the computational complexity of MRSA is *O*(*N* × (2 × *T* × *D*+*T*+1)). The introduction of three improved strategies causes the computational complexity of MRSA to increase slightly compared to RSA. RSA and MRSA can be considered to have similar levels of operating efficiency.

## 4. Experimental Results and Discussion

In this section, we first evaluate various chaotic mapping combination algorithms using benchmark test functions and then determine which chaotic mapping sequence to use in combination with the adaptive reverse learning strategy. The performance of MRSA is then evaluated, and 23 benchmark functions, IEEE CEC2017 benchmark functions, and robot path planning problems are compared with other state-of-the-art algorithms.

### 4.1. Benchmark Test Functions

This section uses 23 benchmark test functions that are commonly found in the literature. These benchmark test functions include seven unimodal functions, six multimodal functions, and ten fixed dimensional functions [55]. Unimodal functions F1–F7 have only one global optimum and are primarily used to test the local exploitation capabilities of the algorithms. The multimodal functions have multiple local minimums and can be used to check the global exploration capability and local optimum avoidance capability of the algorithm. Details of the benchmark test functions are shown in Table 2.

### 4.2. Chaos Mapping Selection Test

The adaptive chaotic reverse learning strategy proposed in this paper combines a chaotic mapping and a reverse learning mechanism. To verify which chaotic mapping is employed, each of the 10 chaotic mappings is combined with a reverse learning mechanism. The MRSA using the chaotic mapping with ID 1 is called MRSA-C1. The rest of the MRSA algorithms using chaotic mappings are named similarly. For a fair comparison, the number of populations was set to 50, and the maximum number of iterations was set to 300 on the same experimental platform. All the algorithms were programmed using MATLAB R2016b, the computer operating system was Windows 10, and the processor was AMD R5 3600 × 16 GB.  Table 3 shows the statistical results of each algorithm run independently 30 times. In presenting the simulation results, “avg” is the average of the best candidate solutions obtained, and “std” is the standard deviation of these values.

As shown in Table 3, MRSA-C1 (Chebyshev map) and MRSA-C9 (Sinusoidal map) outperformed RSA on 10 out of 23 functions. MRSA-C2 (Circle map), MRSA-C3 (Gauss map), MRSA-C5 (Logistic map), MRSA-C6 (Pricewise map), and MRSA-C7 (Sine map) outperformed RSA in 9 functions. MRSA-C4 (Iterative map) outperformed RSA in 12 functions. MRSA-C8 (Singer map) performed better than RSA in 11 functions. MRSA-C10 (Tent map) outperformed RSA on 16 out of 23 functions. Remarkably, all the improved algorithms perform no worse than RSA in at least 22 functions, indicating that the improved strategies proposed in this paper effectively improve the algorithm's performance. Furthermore, the best of the ten chaotic mapping combination algorithms is MRSA-C10. Therefore, the MRSA-C10 algorithm was used to participate in the tests in the comparison that followed.

### 4.3. Performance Comparison Tests of MRSA with Other Advanced Algorithms on 23 Benchmark Functions

To verify the performance of the MRSA algorithm, the modified algorithm was compared with the original RSA [41], HHO [42], EO [43], TSA [44], GWO [36], SSA [45], and WOA [37]. The parameters of all the algorithms were set according to the original paper to ensure the performance of the comparison algorithms, as shown in Table 4. Given that F1–F13 are the multidimensional functions used in this section, the thirteen functions were solved under Dim = 30, 100, 500, and 1000. The means obtained by these algorithms are recorded, as shown in Tables 5–8.

The results in Tables 5–8 show that MRSA achieves better results in most of the functions. Specifically, MRSA obtains satisfactory results for the unimodal functions F1–F7 in both the low and high dimensions. MRSA achieves a stable optimal value of 0 when solving for F1 and F3 and remains so as the dimensionality increases. For the other unimodal functions, HHO outperforms MRSA in solving F7. The unimodal function results show that MRSA outperforms RSA in all the functions, and MRSA does not show a significant decrease in performance as the dimensionality increases, which indicates that the improvement strategy proposed in this paper greatly improves the development capability of RSA. For the variable dimensional multimodal functions F8–F13, MRSA, RSA, HHO, and EO consistently achieve their respective optimal solutions in different dimensions when solving F9–F11. HHO and WOA outperform MRSA in solving F8. MRSA achieves a stable optimal value of 0 when solving for F9 and F11 and remains so as the dimensionality increases. MRSA shows the best performance in solving F12 and F13, outperforming all the compared algorithms. It is worth noting that MRSA does not perform any less than RSA in all the multimodal functions in the different dimensions and has significant improvements in three of the six variable dimensional multimodal functions, which indicates that MRSA has a better global search capability, and the improvement strategy proposed in this paper is well suited to enhance the population diversity and to expand the search range of the population, thus improving the exploration capability of the algorithm.

Table 9 presents the test results when different algorithms solve the fixed dimensional multimodal function. The comparison shows that HHO, EO, and SSA outperform MRSA on F14. For F15–F23, MRSA performs best in all the tested functions. In particular, MRSA provides better solutions in all the test functions compared to RSA. Since fixed-dimension functions are usually used to test the ability of an algorithm to maintain a balance between development and exploration, the above analysis shows that the MRSA proposed in this paper is able to balance the development and exploration capabilities effectively and has a strong local optimum avoidance capability.

The convergence speed and convergence accuracy are important indicators of the performance of the algorithm.  Figure 2 shows the mean convergence curves of MRSA and RSA when solving the test functions in different dimensions. It can be seen that MRSA has a faster convergence speed and a better convergence accuracy in different dimensions. Moreover, the convergence speed and convergence accuracy of MRSA do not decrease much with increasing dimensionality, which indicates that the improvement strategy proposed in this paper can effectively improve the convergence ability of RSA and thus obtain better optimization results.

To analyze the distribution characteristics of each algorithm in the fixed dimensional test function, box plots were drawn based on the results obtained by solving F14–F23, as shown in Figure 3. For each algorithm, the center mark of each box indicates the median of the results of 30 runs, and the bottom and top edges of each box indicate the trivial and quartiles, respectively. “The “+” sign indicates bad values that are not inside the box. As seen from Figure 3, MRSA has no bad values for F17 and F21–F23, which indicates that the distribution of the solutions obtained by MRSA is more concentrated and MRSA is more stable. For the other test functions with some bad values, MRSA outperforms the comparison algorithm in terms of maximum, minimum, and median values, and the distribution of the solutions obtained by MRSA is more concentrated compared to the comparison algorithm. Therefore, MRSA solves the test function with better stability compared to the other comparison algorithms.

Apart from the convergence and stability analysis, to further analyze the experimental results, the Friedman test and Wilcoxon's signed-rank test were used for multiple comparisons in this paper.  Table 10 is the Friedman test showing the average ranking results of each algorithm. The overall ranking value of MRSA is 1.59, which ranks first among all the algorithms. The remaining seven algorithms are ranked as follows: RSA, HHO, EO, WOA, GWO, SSA, and TSA. In solving F1–F13 in different dimensions, MRSA is ranked first, and HHO and RSA are ranked second and third, respectively. For fixed dimensions F14–F23, MRSA, EO, and RSA ranked in the top three. In either case, MRSA ranks better than RSA. The results of Wilcoxon's signed-rank test are shown in Table 11. In the case of F1–F13 (Dim = 30, 100, 500, and 1000), MRSA outperformed EO, TSA, GWO, SSA, WOA, and RSA at the 0.05 significance level, but there was no significant difference between MRSA and HHO. In the case of F14–F23, MRSA outperformed TSA, GWO, WOA, and RSA at the 0.05 significance level, but there was no significant difference between MRSA and HHO, EO, or SSA, which statistically proves that the improvement strategy proposed in this paper can effectively help MRSA balance the exploitation and exploration capabilities and has a better local optimal avoidance ability.

### 4.4. Performance Comparison Tests of MRSA with Other Advanced Algorithms on CEC2017

To further verify the superior performance of the MRSA algorithm, the algorithm was tested using the IEEE CEC2017 [41] single objective test function defined in Table 12. In this section, six recently proposed algorithms were evaluated for comparison with MRSA. These state-of-the-art algorithms are BOA [38], HHO [42], AOA [47], SSA [45], PFA [48], and TDO [46]. For a fair comparison, all the algorithm parameters are set the same as those used by the authors of the original literature, as shown in Table 13. The dimension of the CEC2017 benchmark functions was set to 30 on the same experimental platform.  Table 14 shows the statistical results of each algorithm run independently 51 times.

From the analysis in Table 14, we know that, for the unimodal test function F3, MRSA outperformed all the comparison algorithms, and although MRSA could not stably obtain the optimal solution, it performed the best among all the comparison algorithms, indicating that MRSA has a stronger exploitation ability. For the multipeaked test functions F4–F10, MRSA performs best among the four test functions (F4, F5, F8, and F10), while PFA achieves the best results on F6, F7, and F9, with MRSA ranking second in all cases. The performance of MRSA on the multipeaked functions indicates that the improved algorithm can maintain sufficient population diversity to avoid falling into local optima. For complex and combinatorial functions, each algorithm has its advantages and disadvantages. MRSA obtains optimal solutions on F11–F15, F18-F19, F22, F25, and F28–F30. PFA achieves better solutions on F16-F17, F20, F23-F24, and F26-F27. BOA outperforms the other comparison algorithms on F21. Overall, MRSA achieves the top two results in both the complex and combinatorial functions, better demonstrating the potential of MRSA to solve complex optimization problems in the real world.

To perform a statistical analysis on the performance of MRSA and the six competing algorithms, the Friedman test and Wilcoxon's signed-rank test were used for multiple comparisons in this paper.  Table 15 is the Friedman test results showing the average ranking of each algorithm. The overall ranking value of MRSA is 1.3929, which ranks first among all the algorithms. The remaining six algorithms are ranked as follows: PFA, HHO, TDO, AOA, BOA, and SSA. The results of Wilcoxon's signed-rank test are shown in Table 16. MRSA outperformed BOA, AOA, SSA, PFA, and TDO at the 0.05 significance level, which statistically proves that the improvement strategy proposed in this paper can effectively help MRSA balance the exploitation and exploration capabilities and has a better local optimal avoidance ability.

### 4.5. Robot Path Planning Based on MRSA

To verify the performance of the improved strategy, MRSA is applied to solve the robot path planning in this paper. Each crocodile represents a possible path. It is assumed that there are *N* possible paths, and the dimension *D* is determined by the number of connections from the starting point to the destination point. The environment is modeled using the raster method, and the raster values are used to equate to the obstacles at the location. The robot's working environment is equated to a plane, similar to a lattice effect, and then the feasible and obstacle zones are determined based on the raster values. The grid number 0 is defined as the feasible area, and 1 is defined as the obstacle area. The robot can walk on the grid designated as 0. The cost function for the *i*^th^ crocodile is shown below:

(14) $$\begin{array}{c} \cos t_{i}=\overset{D-1}{\underset{j=1}{\sum }}\sqrt{{\left(x_{j+1}+x_{j}\right)}^{2}+{\left(y_{j+1}+y_{j}\right)}^{2}}\text{,} \end{array}$$

where *j* denotes the *j*^th^ dimension of each crocodile. In robot path planning, the population size is 100, and the number of iterations is 20. RSA [41], HHO [42], and EO [43] are used as competitors. Each algorithm works in a 10 × 10 model, and the optimal route is shown in Figure 4. To eliminate chance, each algorithm was run 10 times, and the mean, optimal, and worst values of each algorithm were recorded. The statistical results of each algorithm are shown in Table 17.

As shown in Figure 4, MRSA has the shortest route, followed by HHO, while EO and RSA are clearly trapped in a local optimum. As seen from Table 17, MRSA is the best among all the algorithms in terms of best cost, mean cost, and worst cost. This indicates that MRSA can consistently provide excellent solutions.  Figure 5 shows the convergence curves of the four algorithms. MRSA has the fastest convergence speed and a higher convergence accuracy. Therefore, the introduction of multiple strategies makes the algorithm more comprehensive in its search, which greatly improves the search capability of MRSA and plans the least costly route.

## 5. Conclusion

This paper proposes a novel variant of the reptile search algorithm, called MRSA. First, the adaptive chaotic reverse learning strategy combines the advantages of the reverse learning mechanism and chaotic mapping to enhance the population diversity. Second, the elite alternative pool strategy balances the exploitation and exploration capabilities by controlling the reference points followed by the population. Finally, the shifted distribution estimation strategy makes full use of the dominant population information to guide the direction of individual evolution, thus improving the performance of RSA. The superiority of MRSA was verified in 23 benchmark functions, IEEE CEC2017 benchmark functions, and robot path planning problems. The experimental results show that the adaptive chaotic reverse learning strategy can effectively improve the population diversity, among which tent mapping is the most effective. The MRSA outperforms the comparison algorithm in terms of convergence accuracy, convergence speed, and stability. The results of the multimodal functions F8–F23 among the 23 benchmark functions show that the elite alternative pool strategy balances algorithm exploitation and exploration effectively and prevents the algorithm from falling into a local optimum. The adaptive chaotic reverse learning strategy enhances the population diversity. The shifted distribution estimation strategy enhances the convergence speed and convergence accuracy of the algorithm by learning information about the dominant populations. In addition, the test results were analyzed using the Friedman test and the Wilcoxon signed-rank test. The statistical results show that MRSA is significantly more effective than the comparison algorithm.

In a subsequent study, we plan to examine the following issues: First, the shifted distribution estimation strategy increases the computational cost of MRSA. Optimizing the algorithm structure and performance needs further investigation and discussion. Second, the capacity and composition of the elite replacement pool need to be further analyzed. Additionally, MRSA can be extended to multiobjective and binary versions. We will consider solving problems in image processing, industry, neural networks, text, and data mining as real-world optimization problems.

## Figures and Tables

**Figure 1:** Flow chart of MRSA.

**Figure 2:** Convergence curves for different dimensional functions.

**Figure 3:** Box plot of different test functions.

**Figure 4:** Path planning diagram: (a) MRSA. (b) RSA. (c) HHO. (d) EO.

**Figure 5:** Convergence curves of four algorithms.

**Algorithm 1:** Pseudocode of the reptile search algorithm (RSA).

**Algorithm 2:** Pseudocode of the MRSA.

**Table 1:** Set of chaotic functions.

ID	Type	Function
1	Chebyshev map	*x*_*i*+1_=cos (*i* cos^−1^(*x*_*i*_))
2	Circle map	*x*_*i*+1_=mod( *x*_*i*_+*b* − (*a*/2*π*) sin (2*πx*_*i*_)), 1), *a*=0.5 *and* *b*=0.2
3	Gauss map	$x_{i+1}=\left\{\begin{array}{c} \;1\;x_{i}=0\;\\ 1/\;\mathrm{mod}\;\left(x_{i},1\right)\;otherwise \end{array}\right.$
4	Iterative map	*x*_*i*+1_=sin (*aπ*/*x*_*i*_), *a*=0.7
5	Logistic map	*x*_*i*+1_=*ax*_*i*_(1 − *x*_*i*_), *a*=4
6	Pricewise map	$x_{i+1}=\left\{\begin{array}{c} x_{i}/p\;0\leq x_{i}<p\\ \left(x_{i}-p\right)/\left(0.5-p\right)\;p\leq x_{i}<0.5\\ \left(1-x_{i}-p\right)/\left(0.5-p\right)\;0.5\leq x_{i}<1-p\\ \left(1-x_{i}\right)/\left(p\right)\;1-p\leq x_{i}<1 \end{array}\right.$
7	Sine map	*x*_*i*+1_=*a*/4 · sin (*πx*_*i*_), *a*=4
8	Singer map	*x*_*i*+1_=*μ*(7.86*x*_*i*_ − 23.32*x*_*i*_^2^+28.75*x*_*i*_^3^ − 13.301875*x*_*i*_^4^), *μ*=1.07
9	Sinusoidal map	*x*_*i*+1_=*ax*_*i*_^2^sin (*πx*_*i*_), *a*=2.3
10	Tent map	$x_{i+1}=\left\{\begin{array}{c} x_{i}/0.7\;x_{i}<0.7\\ 10/3\times \left(1-x_{i}\right)\;x_{i}\geq 0.7 \end{array}\right.$

**Table 2:** The classic benchmark functions (M: multimodal, U: unimodal, S: separable, N: nonseparable, Dim: dimension, Range: limits of search space, Optimum: global optimal value) [55].

Test function	Name	Type	*Dim*	Range	Optimum
*f*_01_(*x*)=*∑*_*i*=1_^*D*^*x*_*i*_^2^	Sphere	US	30	[−100, 100]	0
*f*_02_(*x*)=*∑*_*i*=1_^*D*^|*x*_*i*_|+*∏*_*i*−1_^*D*^|*x*_*i*_|	Schwefel 2.22	UN	30	[−10, 10]	0
*f*_03_(*x*)=*∑*_*i*=1_^*D*^(*∑*_*j*−1_^*D*^*x*_*i*_)^2^	Schwefel 1.2	UN	30	[−100, 100]	0
*f*_04_(*x*)=max_*i*_ {|*x*_*i*_|, 1 ≤ *i* ≤ *D*}	Schwefel 2.21	US	30	[−100, 100]	0
*f*_05_(*x*)=*∑*_*i*=1_^*D*^100(*x*_*i*+1_^2^ − *x*_*i*_^2^)^2^+(*x*_*i*_ − 1)^2^	Rosenbrock	UN	30	[−30, 30]	0
*f*_06_(*x*)=*∑*_*i*=1_^*D*^(⌊*x*_*i*_+0.5⌋)^2^	Step	US	30	[−100, 100]	0
*f*_07_(*x*)=*∑*_*i*=1_^*D*^*ix*_*i*_^4^+random[0,1)	Quartic	US	30	[−1.28,1.28]	0
$f_{08}\left(x\right)=\sum_{i=1}^{D}-x_{i}\sin\left(\sqrt{\left|x_{i}\right|}\right)$	Schwefel 2.26	MS	30	[−500, 500]	-418.9829D
*f*_09_(*x*)=*∑*_*i*=1_^*D*^(*x*_*i*_^2^ − 10 cos (2*πx*_*i*_)+10)	Rastrigin	MS	30	[−5.12, 5.12]	0
$f_{10}\left(x\right)=20+e-20\;\exp\;\left(-0.2\sqrt{1/D\sum_{i=1}^{D}x_{i}^{2}}\right)-\exp\;\left(1/D\sum_{i=1}^{D}\cos\;\left(2\pi x_{i}\right)\right)$	Ackley	MS	30	[−32, 32]	8.8818*e* − 16
$f_{11}\left(x\right)=1/4000\sum_{i=1}^{D}\left(x_{i}^{2}\right)-\left(\prod_{i=1}^{D}\cos\;\left(x_{i}/\sqrt{i}\right)\right)+1$	Griewank	MN	30	[−600, 600]	0
$\begin{array}{c} f_{12}\left(x\right)=\pi /D\left\{10\;\sin\;\left(\pi y_{i}\right)+\sum_{i-1}^{D-1}{\left(y_{i}-1\right)}^{2}\left[1+10\;\sin^{2}\;\left(\pi y_{i+1}\right)\right]+{\left(y_{D}-1\right)}^{2}\right\}\\ +\sum_{i-1}^{D}u\left(x_{i},10,100,4\right)\text{, where}y_{i}=1+x_{i}+\;u\left(x_{i},a,k,m\right)=\left\{\begin{array}{c} k{\left(x_{i}-a\right)}^{m}\;x_{i}>a\\ 0-a<x_{i}<a\\ k{\left(-x_{i}-a\right)}^{m}x_{i}<a \end{array}\right. \end{array}$	Penalized	MN	30	[−50, 50]	0
$\begin{array}{c} f_{13}\left(x\right)=0.1\;\left(\sin^{2}\right.\;\left(3\pi x_{i}\right)+\sum_{i=1}^{D}{\left(x_{i}-1\right)}^{2}\left[1+\sin^{2}\;\left(3\pi x_{i}\right)\right]+{\left(x_{D}-1\right)}^{2}1+\\ \;\sin^{2}\;\left.\left.\left(2\pi x_{D}\right)\right]\right\}+\sum_{i-1}^{D}u\left(x_{i},5,100,4\right) \end{array}$	Penalized2	MN	30	[−50, 50]	0
*f*_14_(*x*)=(1/500+*∑*_*j*=1_^25^1/*j*+*∑*_*i*=1_^2^(*x*_*i*_ − *a*_*ij*_)^6^)^−1^	Foxholes	MS	2	[−65.53,65.53]	0.998004
*f*_15_(*x*)=*∑*_*i*=1_^11^(*a*_*i*_ − *x*_1_(*b*_*i*_^2^+*b*_*i*_*x*_2_)/(*b*_*i*_^2^+*b*_*i*_*x*_3_+*x*_4_))^−1^	Kowalik	MS	4	[−5, 5]	0.0003075
*f*_16_(*x*)=4*x*_1_^2^ − 2.1*x*_1_^4^+1/3*x*_1_^6^+*x*_1_*x*_2_ − 4*x*_2_^2^+*x*_2_^4^	Six-hump camel back	MN	2	[−5, 5]	−1.03163
*f*_17_(*x*)=(*x*_2_ − 5.1/4*π*^2^*∗x*_1_^2^+5/*π∗x*_1_ − 6)^2^+10(1 − 1/8*π*)cos*x*_1_+10	Branin	MS	2	[−5, 10] × [0, 15]	0.398
$\begin{array}{c} f_{18}\left(x\right)=\left[1+{\left(x_{1}+x_{2}+1\right)}^{2}\left(19-14x_{1}+3x_{1}^{2}-14x_{2}+6x_{1}x_{2}+3x_{2}^{2}\right)\right]\\ \times \left[30+{\left(2x_{1}-3x_{2}\right)}^{2}\left(18-32x_{1}+12x_{1}^{2}+48x_{2}-36x_{1}x_{2}+27x_{2}^{2}\right)\right] \end{array}$	Goldstein-Price	MN	2	[−5, 5]	3
*f*_19_(*x*)=−*∑*_*i*=1_^4^(*c*_*i*_exp − (*∑*_*j*−1_^3^*a*_*ij*_(*x*_*j*_ − *p*_*ij*_^2^))	Hartman 3	MN	3	[0, 1]	−3.8628
*f*_20_(*x*)=−*∑*_*i*=1_^4^(*c*_*i*_exp − (*∑*_*j*−1_^6^*a*_*ij*_(*x*_*j*_ − *p*_*ij*_^2^))	Hartman 6	MN	6	[0, 1]	−3.32
*f*_21_(*x*)=−*∑*_*i*=1_^5^[(*X* − *a*_*i*_)(*X* − *a*_*i*_)^*T*^+*c*_*i*_]^−1^	Langermann 5	MN	4	[0, 10]	−10.1532
*f*_22_(*x*)=−*∑*_*i*=1_^7^[(*X* − *a*_*i*_)(*X* − *a*_*i*_)^*T*^+*c*_*i*_]^−1^	Langermann 7	MN	4	[0, 10]	−10.4029
*f*_23_(*x*)=−*∑*_*i*=1_^10^[(*X* − *a*_*i*_)(*X* − *a*_*i*_)^*T*^+*c*_*i*_]^−1^	Langermann 10	MN	4	[0, 10]	−10.5364

**Table 3:** Results of 10 chaotic maps on all benchmark functions.

Function	Index	MRSA-C1	MRSA-C2	MRSA-C3	MRSA-C4	MRSA-C5	MRSA-C6	MRSA-C7	MRSA-C8	MRSA-C9	MRSA-C10	RSA [41]
F1	Mean	2.51*E* − 155	8.11*E* − 219	5.13*E* − 226	3.37*E* − 157	4.35*E* − 219	3.96*E* − 207	1.73*E* − 223	4.11*E* − 224	6.09*E* − 226	8.09*E* − 260	2.48*E* − 65
	Std	1.37*E* − 154	0.00*E* + 00	0.00*E* + 00	1.84*E* − 156	0.00*E* + 00	0.00*E* + 00	0.00*E* + 00	0.00*E* + 00	0.00*E* + 00	0.00*E* + 00	1.36*E* − 64
	Rank	10	7	2	9	6	8	5	4	3	**1**	11

F2	Mean	8.71*E* − 82	2.94*E* − 111	4.34*E* − 108	5.97*E* − 78	2.47*E* − 109	7.33*E* − 109	2.41*E* − 114	5.55*E* − 111	7.68*E* − 104	3.33*E* − 136	7.60*E* − 32
	Std	3.52*E* − 81	1.61*E* − 110	1.66*E* − 107	2.87*E* − 77	1.29*E* − 108	3.33*E* − 108	1.04*E* − 113	2.35*E* − 110	4.21*E* − 103	1.82*E* − 135	2.36*E* − 31
	Rank	9	3	7	10	5	6	2	4	8	**1**	11

F3	Mean	7.40*E* − 113	9.15*E* − 192	7.28*E* − 180	2.82*E* − 117	2.94*E* − 186	7.00*E* − 187	6.73*E* − 185	1.23*E* − 182	1.34*E* − 190	1.54*E* − 247	6.80*E* − 43
	Std	4.06*E* − 112	0.00*E* + 00	0.00*E* + 00	1.55*E* − 116	0.00*E* + 00	0.00*E* + 00	0.00*E* + 00	0.00*E* + 00	0.00*E* + 00	0.00*E* + 00	3.72*E* − 42
	Rank	10	2	8	9	5	4	6	7	3	**1**	11

F4	Mean	5.72*E* − 80	3.02*E* − 106	1.24*E* − 104	5.63*E* − 80	4.65*E* − 109	1.13*E* − 107	2.23*E* − 108	8.95*E* − 111	9.60*E* − 111	6.19*E* − 137	5.88*E* − 35
	Std	2.84*E* − 79	1.65*E* − 105	6.79*E* − 104	2.18*E* − 79	2.53*E* − 108	5.94*E* − 107	1.22*E* − 107	3.20*E* − 110	3.57*E* − 110	3.32*E* − 136	3.22*E* − 34
	Rank	10	7	8	9	4	6	5	2	3	**1**	11

F5	Mean	1.80*E* − 07	4.62*E* − 07	3.64*E* − 07	4.71*E* − 08	4.50*E* − 07	3.54*E* − 07	2.61*E* − 07	3.13*E* − 07	5.97*E* − 07	1.02*E* − 06	4.34*E* − 05
	Std	3.25*E* − 07	1.16*E* − 06	1.17*E* − 06	9.59*E* − 08	2.05*E* − 06	1.47*E* − 06	5.61*E* − 07	5.42*E* − 07	1.68*E* − 06	2.49*E* − 06	6.90*E* − 05
	Rank	2	8	6	**1**	7	5	3	4	9	10	11

F6	Mean	4.18*E* − 12	1.24*E* − 12	1.28*E* − 12	5.05*E* − 12	4.65*E* − 12	8.84*E* − 13	6.78*E* − 13	1.06*E* − 12	1.07*E* − 12	5.88*E* − 13	1.54*E* − 09
	Std	1.22*E* − 11	2.70*E* − 12	3.04*E* − 12	2.36*E* − 11	2.21*E* − 11	1.42*E* − 12	2.25*E* − 12	1.90*E* − 12	2.74*E* − 12	1.04*E* − 12	3.30*E* − 09
	Rank	8	6	7	10	9	3	2	4	5	**1**	11

F7	Mean	3.84*E* − 04	2.66*E* − 04	1.92*E* − 04	3.40*E* − 04	2.71*E* − 04	2.56*E* − 04	2.21*E* − 04	2.02*E* − 04	2.54*E* − 04	1.81*E* − 04	5.54*E* − 04
	Std	3.47*E* − 04	1.86*E* − 04	1.98*E* − 04	2.65*E* − 04	1.56*E* − 04	2.01*E* − 04	2.36*E* − 04	1.47*E* − 04	2.30*E* − 04	1.55*E* − 04	5.97*E* − 04
	Rank	10	7	2	9	8	6	4	3	5	**1**	11

F8	Mean	−7.63*E* + 03	−8.97*E* + 03	−8.67*E* + 03	−8.00*E* + 03	−8.39*E* + 03	−8.22*E* + 03	−8.96*E* + 03	−9.29*E* + 03	−8.99*E* + 03	−8.44*E* + 03	−8.29*E* + 03
	Std	7.50*E* + 02	1.73*E* + 03	1.64*E* + 03	1.04*E* + 03	9.94*E* + 02	1.02*E* + 03	1.45*E* + 03	1.74*E* + 03	1.47*E* + 03	5.81*E* + 02	5.78*E* + 02
	Rank	11	3	5	10	7	9	4	**1**	2	6	8

F9	Mean	0.00*E* + 00	0.00*E* + 00	0.00*E* + 00	0.00*E* + 00	0.00*E* + 00	0.00*E* + 00	0.00*E* + 00	0.00*E* + 00	0.00*E* + 00	0.00*E* + 00	0.00*E* + 00
	Std	0.00*E* + 00	0.00*E* + 00	0.00*E* + 00	0.00*E* + 00	0.00*E* + 00	0.00*E* + 00	0.00*E* + 00	0.00*E* + 00	0.00*E* + 00	0.00*E* + 00	0.00*E* + 00
	Rank	**1**	**1**	**1**	**1**	**1**	**1**	**1**	**1**	**1**	**1**	**1**

F10	Mean	8.88*E* − 16	8.88*E* − 16	8.88*E* − 16	8.88*E* − 16	8.88*E* − 16	8.88*E* − 16	8.88*E* − 16	8.88*E* − 16	8.88*E* − 16	8.88*E* − 16	8.88*E* − 16
	Std	0.00*E* + 00	0.00*E* + 00	0.00*E* + 00	0.00*E* + 00	0.00*E* + 00	0.00*E* + 00	0.00*E* + 00	0.00*E* + 00	0.00*E* + 00	0.00*E* + 00	0.00*E* + 00
	Rank	**1**	**1**	**1**	**1**	**1**	**1**	**1**	**1**	**1**	**1**	**1**

F11	Mean	0.00*E* + 00	0.00*E* + 00	0.00*E* + 00	0.00*E* + 00	0.00*E* + 00	0.00*E* + 00	0.00*E* + 00	0.00*E* + 00	0.00*E* + 00	0.00*E* + 00	0.00*E* + 00
	Std	0.00*E* + 00	0.00*E* + 00	0.00*E* + 00	0.00*E* + 00	0.00*E* + 00	0.00*E* + 00	0.00*E* + 00	0.00*E* + 00	0.00*E* + 00	0.00*E* + 00	0.00*E* + 00
	Rank	**1**	**1**	**1**	**1**	**1**	**1**	**1**	**1**	**1**	**1**	**1**

F12	Mean	6.09*E* − 13	4.86*E* − 13	6.84*E* − 13	2.35*E* − 13	1.55*E* − 12	3.62*E* − 13	3.36*E* − 13	2.93*E* − 13	5.16*E* − 13	6.21*E* − 13	4.51*E* − 11
	Std	2.06*E* − 12	6.87*E* − 13	1.87*E* − 12	4.26*E* − 13	5.95*E* − 12	6.65*E* − 13	6.92*E* − 13	5.74*E* − 13	1.16*E* − 12	1.59*E* − 12	1.95*E* − 10
	Rank	7	5	9	**1**	10	4	3	2	6	8	11

F13	Mean	5.56*E* − 12	2.44*E* − 11	1.86*E* − 11	7.55*E* − 12	1.54*E* − 11	1.41*E* − 11	1.00*E* − 11	8.05*E* − 12	1.27*E* − 11	2.79*E* − 11	1.84*E* − 09
	Std	1.56*E* − 11	6.58*E* − 11	4.90*E* − 11	2.39*E* − 11	7.35*E* − 11	2.19*E* − 11	2.03*E* − 11	2.37*E* − 11	2.74*E* − 11	1.11*E* − 10	6.87*E* − 09
	Rank	**1**	9	8	2	7	6	4	3	5	10	11

F14	Mean	1.06*E* + 00	1.79*E* + 00	1.59*E* + 00	1.52*E* + 00	1.62*E* + 00	2.17*E* + 00	1.46*E* + 00	2.76*E* + 00	1.20*E* + 00	9.98*E* − 01	8.98*E* + 00
	Std	3.62*E* − 01	1.90*E* + 00	1.86*E* + 00	1.85*E* + 00	1.90*E* + 00	2.97*E* + 00	1.83*E* + 00	3.68*E* + 00	6.05*E* − 01	1.54*E* − 16	5.34*E* + 00
	Rank	2	8	6	5	7	9	4	10	3	**1**	11

F15	Mean	3.07*E* − 04	3.07*E* − 04	3.07*E* − 04	3.07*E* − 04	3.07*E* − 04	3.07*E* − 04	3.07*E* − 04	3.07*E* − 04	3.07*E* − 04	3.07*E* − 04	3.35*E* − 04
	Std	2.19*E* − 11	3.38*E* − 11	1.30*E* − 10	2.78*E* − 10	1.02*E* − 10	7.23*E* − 11	6.56*E* − 12	2.16*E* − 12	5.91*E* − 12	7.98*E* − 12	1.03*E* − 04
	Rank	5	6	9	10	8	7	4	**1**	2	3	11

F16	Mean	−1.03*E* + 00	−1.03*E* + 00	−1.03*E* + 00	−1.03*E* + 00	−1.03*E* + 00	−1.03*E* + 00	−1.03*E* + 00	−1.03*E* + 00	−1.03*E* + 00	−1.03*E* + 00	−1.03*E* + 00
	Std	5.98*E* − 16	5.68*E* − 16	6.12*E* − 16	5.76*E* − 16	5.61*E* − 16	5.22*E* − 16	5.53*E* − 16	5.83*E* − 16	5.68*E* − 16	5.68*E* − 16	5.68*E* − 16
	Rank	**1**	**1**	**1**	**1**	**1**	**1**	**1**	**1**	**1**	**1**	**1**

F17	Mean	3.98*E* − 01	3.98*E* − 01	3.98*E* − 01	3.98*E* − 01	3.98*E* − 01	3.98*E* − 01	3.98*E* − 01	3.98*E* − 01	3.98*E* − 01	3.98*E* − 01	3.98*E* − 01
	Std	0.00*E* + 00	0.00*E* + 00	0.00*E* + 00	0.00*E* + 00	0.00*E* + 00	0.00*E* + 00	0.00*E* + 00	0.00*E* + 00	0.00*E* + 00	0.00*E* + 00	0.00*E* + 00
	Rank	**1**	**1**	**1**	**1**	**1**	**1**	**1**	**1**	**1**	**1**	**1**

F18	Mean	4.80*E* + 00	3.00*E* + 00	3.00*E* + 00	3.00*E* + 00	3.00*E* + 00	3.00*E* + 00	3.00*E* + 00	3.00*E* + 00	3.00*E* + 00	3.00*E* + 00	6.60*E* + 00
	Std	6.85*E* + 00	1.62*E* − 15	1.51*E* − 15	1.79*E* − 15	1.95*E* − 15	1.74*E* − 15	7.71*E* − 11	2.00*E* − 15	1.10*E* − 15	1.28*E* − 15	9.34*E* + 00
	Rank	10	6	2	4	8	4	9	6	**1**	2	11

F19	Mean	−3.86*E* + 00	−3.86*E* + 00	−3.86*E* + 00	−3.86*E* + 00	−3.86*E* + 00	−3.86*E* + 00	−3.86*E* + 00	−3.86*E* + 00	−3.86*E* + 00	−3.86*E* + 00	−3.86*E* + 00
	Std	2.37*E* − 15	2.42*E* − 15	2.43*E* − 15	2.34*E* − 15	2.46*E* − 15	2.42*E* − 15	2.45*E* − 15	2.46*E* − 15	2.46*E* − 15	2.39*E* − 15	2.42*E* − 15
	Rank	**1**	**1**	**1**	**1**	**1**	**1**	**1**	**1**	**1**	**1**	**1**

F20	Mean	−3.27*E* + 00	−3.27*E* + 00	−3.26*E* + 00	−3.30*E* + 00	−3.28*E* + 00	−3.27*E* + 00	−3.28*E* + 00	−3.27*E* + 00	−3.27*E* + 00	−3.27*E* + 00	−3.28*E* + 00
	Std	5.92*E* − 02	5.99*E* − 02	6.03*E* − 02	4.84*E* − 02	5.70*E* − 02	5.99*E* − 02	5.83*E* − 02	5.92*E* − 02	5.99*E* − 02	5.92*E* − 02	5.83*E* − 02
	Rank	5	8	11	**1**	2	8	3	5	8	5	3

F21	Mean	−1.02*E* + 01	−1.02*E* + 01	−1.02*E* + 01	−1.02*E* + 01	−1.02*E* + 01	−1.02*E* + 01	−1.02*E* + 01	−1.02*E* + 01	−1.02*E* + 01	−1.02*E* + 01	−8.96*E* + 00
	Std	5.63*E* − 15	5.56*E* − 15	5.51*E* − 15	5.44*E* − 15	5.78*E* − 15	5.56*E* − 15	5.63*E* − 15	5.46*E* − 15	5.55*E* − 15	5.46*E* − 15	2.19*E* + 00
	Rank	**1**	**1**	**1**	**1**	**1**	**1**	**1**	**1**	**1**	**1**	11

F22	Mean	−1.04*E* + 01	−1.04*E* + 01	−1.04*E* + 01	−1.04*E* + 01	−1.04*E* + 01	−1.04*E* + 01	−1.04*E* + 01	−1.04*E* + 01	−1.04*E* + 01	−1.04*E* + 01	−9.16*E* + 00
	Std	8.73*E* − 16	8.73*E* − 16	8.08*E* − 16	4.66*E* − 16	8.08*E* − 16	8.73*E* − 16	7.38*E* − 16	9.33*E* − 16	7.38*E* − 16	1.09*E* − 15	2.29*E* + 00
	Rank	**1**	**1**	**1**	**1**	**1**	**1**	**1**	**1**	**1**	**1**	11

F23	Mean	−1.05*E* + 01	−1.05*E* + 01	−1.05*E* + 01	−1.05*E* + 01	−1.05*E* + 01	−1.05*E* + 01	−1.05*E* + 01	−1.05*E* + 01	−1.05*E* + 01	−1.05*E* + 01	−9.45*E* + 00
	Std	2.11*E* − 15	2.24*E* − 15	1.92*E* − 15	1.78*E* − 15	1.75*E* − 15	2.03*E* − 15	1.75*E* − 15	2.09*E* − 15	2.01*E* − 15	1.78*E* − 15	2.20*E* + 00
	Rank	**1**	**1**	**1**	**1**	**1**	**1**	**1**	**1**	**1**	**1**	11

**Table 4:** Parameter setting for comparison algorithm.

Algorithm	Parameters
HHO [42]	*β*=1.5, *E*_0_ ∈ [−1,1]
EO [43]	*a*_1_=2, *a*_2_=1
TSA [44]	*P*_max_=4, *P*_min_=1
GWO [36]	*a*=2 (linearly decreased over iterations)
SSA [45]	*c*_1_=*rand*, *c*_2_=*rand*
WOA [37]	*a*_1_=2 (linearly decreased over iterations)
RSA [41]	*α*=0.1, *β*=0.1

**Table 5:** Test results of different algorithms for F1–F13 (Dim = 30).

30D	MRSA	HHO [42]	EO [43]	TSA [44]	GWO [36]	SSA [45]	WOA [37]	RSA [41]
F1	**0.00E + 00**	1.06*E* − 187	1.68*E* − 72	6.24*E* − 27	2.09*E* − 34	1.14*E* − 02	2.32*E* − 166	2.10*E* − 182
F2	**1.29E − 248**	4.21*E* − 100	2.03*E* − 42	1.12*E* − 17	6.77*E* − 21	1.43*E* + 01	5.11*E* − 107	8.28*E* − 93
F3	**0.00E + 00**	5.81*E* − 135	5.43*E* − 06	7.48*E* + 02	7.43*E* − 01	1.91*E* + 04	7.02*E* + 05	6.13*E* − 116
F4	**7.53E − 256**	3.88*E* − 96	1.87*E* − 11	2.95*E* + 01	6.86*E* − 05	2.05*E* + 01	7.27*E* + 01	4.55*E* − 109
F5	**3.89E − 07**	3.67*E* − 03	9.41*E* + 01	9.80*E* + 01	9.72*E* + 01	6.74*E* + 02	9.73*E* + 01	4.69*E* − 05
F6	**4.26E − 10**	3.74*E* − 05	9.21*E* − 02	1.36*E* + 01	7.86*E* + 00	1.64*E* − 02	5.45*E* − 01	4.76*E* − 08
F7	6.11*E* − 05	**4.18E − 05**	7.93*E* − 04	1.32*E* − 02	1.76*E* − 03	8.03*E* − 01	8.11*E* − 04	2.38*E* − 04
F8	−3.60*E* + 04	**−4.19E + 04**	−2.92*E* + 04	−1.42*E* + 04	−1.61*E* + 04	−2.38*E* + 04	−4.01*E* + 04	−2.47*E* + 04
F9	**0.00E + 00**	**0.00E + 00**	**0.00E + 00**	9.12*E* + 02	2.23*E* − 01	1.34*E* + 02	3.79*E* − 15	**0.00E + 00**
F10	**8.88E − 16**	**8.88E − 16**	7.99*E* − 15	4.96*E* − 14	6.97*E* − 14	5.14*E* + 00	4.91*E* − 15	**8.88E − 16**
F11	**0.00E + 00**	**0.00E + 00**	**0.00E + 00**	2.04*E* − 03	2.57*E* − 03	1.01*E* − 01	**0.00E + 00**	**0.00E + 00**
F12	**9.70E − 12**	3.36*E* − 07	4.13*E* − 04	1.01*E* + 01	1.83*E* − 01	1.15*E* + 01	5.96*E* − 03	3.51*E* − 10
F13	**3.42E − 10**	1.51*E* − 05	2.30*E* + 00	1.17*E* + 01	5.60*E* + 00	1.61*E* + 02	7.29*E* − 01	2.92*E* − 08

**Table 6:** Test results of different algorithms for F1–F13 (Dim = 100).

100D	MRSA	HHO [42]	EO [43]	TSA [44]	GWO [36]	SSA [45]	WOA [37]	RSA [41]
F1	**0.00E + 00**	3.63*E* − 193	7.51*E* − 73	1.25*E* − 27	3.22*E* − 34	1.03*E* − 02	4.14*E* − 166	9.57*E* − 183
F2	**3.08E − 251**	4.29*E* − 100	2.29*E* − 42	1.10*E* − 17	7.27*E* − 21	1.23*E* + 01	3.27*E* − 106	2.05*E* − 101
F3	**0.00E + 00**	1.47*E* − 142	2.51*E* − 06	1.03*E* + 03	9.92*E* − 01	2.04*E* + 04	6.76*E* + 05	1.78*E* − 122
F4	**1.01E − 254**	4.63*E* − 93	2.04*E* − 11	2.98*E* + 01	4.34*E* − 04	2.07*E* + 01	7.47*E* + 01	8.33*E* − 93
F5	**1.86E − 07**	4.44*E* − 03	9.39*E* + 01	9.81*E* + 01	9.72*E* + 01	5.52*E* + 02	9.72*E* + 01	3.67*E* − 05
F6	**2.52E − 11**	2.76*E* − 05	1.56*E* − 01	1.38*E* + 01	7.65*E* + 00	6.61*E* − 03	5.85*E* − 01	4.85*E* − 08
F7	7.56*E* − 05	**3.24E − 05**	8.65*E* − 04	1.63*E* − 02	1.75*E* − 03	7.38*E* − 01	1.66*E* − 03	2.54*E* − 04
F8	−3.36*E* + 04	**−4.19E + 04**	−2.92*E* + 04	−1.45*E* + 04	−1.62*E* + 04	−2.38*E* + 04	−3.72*E* + 04	−2.50*E* + 04
F9	**0.00E + 00**	**0.00E + 00**	**0.00E + 00**	9.28*E* + 02	4.94*E* − 01	1.29*E* + 02	3.79*E* − 15	**0.00E + 00**
F10	**8.88E − 16**	**8.88E − 16**	7.88*E* − 15	8.02*E* − 02	6.93*E* − 14	5.04*E* + 00	4.56*E* − 15	**8.88E − 16**
F11	**0.00E + 00**	**0.00E + 00**	**0.00E + 00**	2.25*E* − 03	1.61*E* − 03	1.07*E* − 01	2.41*E* − 03	**0.00E + 00**
F12	**9.43E − 13**	2.55*E* − 07	2.02*E* − 04	9.78*E* + 00	1.80*E* − 01	1.13*E* + 01	5.40*E* − 03	7.39*E* − 10
F13	**2.25E − 10**	1.12*E* − 05	2.07*E* + 00	1.19*E* + 01	5.72*E* + 00	1.57*E* + 02	6.03*E* − 01	1.13*E* − 08

**Table 7:** Test results of different algorithms for F1–F13 (Dim = 500).

500D	MRSA	HHO [42]	EO [43]	TSA [44]	GWO [36]	SSA [45]	WOA [37]	RSA [41]
F1	**0.00E + 00**	2.61*E* − 195	1.13*E* − 72	7.72*E* − 28	1.82*E* − 34	6.70*E* − 03	1.27*E* − 165	7.20*E* − 175
F2	**1.13E − 250**	3.07*E* − 99	2.64*E* − 42	9.40*E* − 18	7.22*E* − 21	1.31*E* + 01	1.54*E* − 108	7.77*E* − 103
F3	**0.00E + 00**	3.88*E* − 121	3.93*E* − 05	5.72*E* + 02	3.37*E* − 01	1.67*E* + 04	7.11*E* + 05	5.41*E* − 136
F4	**1.47E − 259**	3.18*E* − 98	9.92*E* − 03	3.19*E* + 01	6.68*E* − 05	2.01*E* + 01	8.02*E* + 01	2.27*E* − 105
F5	**4.99E − 07**	3.65*E* − 03	9.40*E* + 01	9.83*E* + 01	9.71*E* + 01	5.06*E* + 02	9.72*E* + 01	3.68*E* − 05
F6	**8.10E − 11**	6.80*E* − 05	1.33*E* − 01	1.36*E* + 01	7.81*E* + 00	7.64*E* − 03	5.83*E* − 01	5.17*E* − 08
F7	7.12*E* − 05	**5.01E − 05**	7.65*E* − 04	1.54*E* − 02	1.62*E* − 03	7.27*E* − 01	1.79*E* − 03	2.23*E* − 04
F8	−3.40*E* + 04	**−4.19E + 04**	−2.90*E* + 04	−1.44*E* + 04	−1.63*E* + 04	−2.45*E* + 04	−3.99*E* + 04	−2.46*E* + 04
F9	**0.00E + 00**	**0.00E + 00**	**0.00E + 00**	8.69*E* + 02	7.10*E* − 02	1.37*E* + 02	**0.00E + 00**	**0.00E + 00**
F10	**8.88E − 16**	**8.88E − 16**	7.99*E* − 15	1.78*E* − 01	6.98*E* − 14	4.97*E* + 00	3.85*E* − 15	**8.88E − 16**
F11	**0.00E + 00**	**0.00E + 00**	**0.00E + 00**	3.16*E* − 03	3.28*E* − 04	1.10*E* − 01	**0.00E + 00**	**0.00E + 00**
F12	**6.72E − 12**	3.29*E* − 07	9.68*E* − 04	1.03*E* + 01	1.85*E* − 01	1.15*E* + 01	5.97*E* − 03	2.03*E* − 10
F13	**9.35 ** *E* − **11**	8.81*E* − 06	2.23*E* + 00	1.17*E* + 01	5.63*E* + 00	1.55*E* + 02	6.80*E* − 01	3.90*E* − 08

**Table 8:** Test results of different algorithms for F1–F13 (Dim = 1000).

1000D	MRSA	HHO [42]	EO [43]	TSA [44]	GWO [36]	SSA [45]	WOA [37]	RSA [41]
F1	**0.00E + 00**	7.31*E* − 188	6.27*E* − 56	3.27*E* − 08	5.24*E* − 10	1.19*E* + 05	8.86*E* − 163	1.80*E* − 186
F2	**2.83E − 236**	6.65*E* − 99	2.70*E* − 33	3.03*E* − 07	2.64*E* − 05	8.48*E* + 02	2.51*E* − 105	1.52*E* − 86
F3	**0.00E + 00**	6.88*E* − 83	2.98*E* + 04	3.99*E* + 06	5.80*E* + 05	2.34*E* + 06	1.03*E* + 08	1.38*E* − 157
F4	**4.64E − 266**	1.59*E* − 94	8.56*E* + 01	9.95*E* + 01	7.27*E* + 01	3.63*E* + 01	8.08*E* + 01	1.09*E* − 97
F5	**5.37E − 05**	3.62*E* − 02	9.96*E* + 02	9.91*E* + 03	9.97*E* + 02	3.03*E* + 07	9.91*E* + 02	4.88*E* − 04
F6	**4.95E − 07**	3.61*E* − 04	1.69*E* + 02	2.06*E* + 02	2.02*E* + 02	1.18*E* + 05	2.32*E* + 01	5.34*E* − 06
F7	7.24*E* − 05	**5.54E − 05**	1.59*E* − 03	1.92*E* + 00	1.30*E* − 02	4.38*E* + 02	1.67*E* − 03	3.87*E* − 04
F8	−3.82*E* + 05	**−4.19E + 05**	−1.57*E* + 05	−4.98*E* + 04	−1.08*E* + 05	−1.30*E* + 05	−4.04*E* + 05	−1.60*E* + 05
F9	**0.00E + 00**	**0.00E + 00**	**0.00E + 00**	1.10*E* + 04	1.09*E* + 01	5.61*E* + 03	1.21*E* − 13	**0.00E + 00**
F10	**8.88E − 16**	**8.88E − 16**	1.07*E* − 14	7.83*E* − 06	7.54*E* − 07	1.29*E* + 01	3.97*E* − 15	**8.88E − 16**
F11	**0.00E + 00**	**0.00E + 00**	8.88*E* − 17	1.77*E* − 02	3.16*E* − 03	1.08*E* + 03	3.70*E* − 18	**0.00E + 00**
F12	**1.75E − 10**	1.50*E* − 07	5.43*E* − 01	3.82*E* + 06	8.37*E* − 01	6.96*E* + 04	1.89*E* − 02	1.82*E* − 09
F13	**8.09E − 08**	4.45*E* − 05	9.90*E* + 01	4.51*E* + 05	9.50*E* + 01	1.41*E* + 07	1.04*E* + 01	7.07*E* − 07

**Table 9:** Test results of different algorithms for F14–F23.

	MRSA	HHO [42]	EO [43]	TSA [44]	GWO [36]	SSA [45]	WOA [37]	RSA [41]
F14	1.13*E* + 00	1.06*E* + 00	**9.98E − 01**	8.28*E* + 00	3.00*E* + 00	**9.98E − 01**	1.78*E* + 00	5.34*E* + 00
F15	**3.07E − 04**	3.46*E* − 04	3.68*E* − 03	5.17*E* − 03	3.04*E* − 03	7.66*E* − 04	6.61*E* − 04	3.21*E* − 04
F16	**−1.03E + 00**	**−1.03E + 00**	**−1.03E + 00**	**−1.03E + 00**	**−1.03E + 00**	**−1.03E + 00**	**−1.03E + 00**	**−1.03E + 00**
F17	**3.98E − 01**	**3.98E − 01**	**3.98E − 01**	**3.98E − 01**	**3.98E − 01**	**3.98E − 01**	**3.98E − 01**	**3.98E − 01**
F18	**3.00E + 00**	**3.00E + 00**	**3.00E + 00**	8.40*E* + 00	**3.00E + 00**	**3.00E + 00**	**3.00E + 00**	5.70*E* + 00
F19	**−3.86E + 00**	**−3.86E + 00**	**−3.86E + 00**	**−3.86E + 00**	**−3.86E + 00**	**−3.86E + 00**	**−3.86E + 00**	**−3.86E + 00**
F20	**−3.27E + 00**	−3.17*E* + 00	−3.26*E* + 00	−3.24*E* + 00	**−3.27E + 00**	−3.22*E* + 00	−3.22*E* + 00	−3.26*E* + 00
F21	**−1.02E + 01**	−5.22*E* + 00	−9.05*E* + 00	−6.23*E* + 00	−9.48*E* + 00	−8.47*E* + 00	−9.56*E* + 00	−9.81*E* + 00
F22	**−1.04E + 01**	−5.44*E* + 00	**−1.04E + 01**	−7.62*E* + 00	−1.00*E* + 01	−9.97*E* + 00	−9.08*E* + 00	**−1.04E + 01**
F23	**−1.05E + 01**	−5.67*E* + 00	−9.91*E* + 00	−6.05*E* + 00	−1.04*E* + 01	−1.04*E* + 01	−9.64*E* + 00	−1.04*E* + 01

**Table 10:** The Friedman test results for different algorithms.

Function	Type	MRSA	HHO [42]	EO [43]	TSA [44]	GWO [36]	SSA [45]	WOA [37]	RSA [41]
F1–F13	Dim = 30	1.58	2.42	4.19	7.00	6.08	7.23	4.77	2.73
	Dim = 100	1.54	2.38	4.15	7.08	5.85	7.23	5.08	2.69
	Dim = 500	1.62	2.62	4.31	7.15	5.77	7.23	4.69	2.62
	Dim = 1000	1.50	2.42	4.88	7.23	5.92	7.23	4.31	2.50

F14–F23	Fixed dim	1.75	5.80	3.05	7.10	5.20	4.20	5.50	3.40

All cases		**1.59**	3.00	4.17	7.11	5.79	6.74	4.84	2.76

**Table 11:** The Wilcoxon signed-rank test results for different algorithms.

Functions type	Comparison	*p* value	*α* = 0.05
F1–F13 (Dim = 30)	MRSA versus HHO [42]	**0.182338**	No
	MRSA versus EO [43]	0.001871	Yes
	MRSA versus TSA [44]	0.001306	Yes
	MRSA versus GWO [36]	0.001306	Yes
	MRSA versus SSA [45]	0.001306	Yes
	MRSA versus WOA [37]	0.02537	Yes
	MRSA versus RSA [41]	0.002873	Yes

F1–F13 (Dim = 100)	MRSA versus HHO [42]	**0.209427**	No
	MRSA versus EO [43]	0.001871	Yes
	MRSA versus TSA [44]	0.001306	Yes
	MRSA versus GWO [36]	0.001306	Yes
	MRSA versus SSA [45]	0.001306	Yes
	MRSA versus WOA [37]	0.017496	Yes
	MRSA versus RSA [41]	0.002873	Yes

F1–F13 (Dim = 500)	MRSA versus HHO [42]	**0.182338**	No
	MRSA versus EO [43]	0.001871	Yes
	MRSA versus TSA [44]	0.001306	Yes
	MRSA versus GWO [36]	0.001306	Yes
	MRSA versus SSA [45]	0.001306	Yes
	MRSA versus WOA [37]	0.02313	Yes
	MRSA versus RSA [41]	0.002873	Yes

F1–F13 (Dim = 1000)	MRSA versus HHO [42]	**0.157939**	No
	MRSA versus EO [43]	0.001944	Yes
	MRSA versus TSA [44]	0.001306	Yes
	MRSA versus GWO [36]	0.001306	Yes
	MRSA versus SSA [45]	0.001306	Yes
	MRSA versus WOA [37]	0.017496	Yes
	MRSA versus RSA [41]	0.002873	Yes

F14–F23	MRSA versus HHO [42]	**0.083131**	No
	MRSA versus EO [43]	**0.192518**	No
	MRSA versus TSA [44]	0.010862	Yes
	MRSA versus GWO [36]	0.032969	Yes
	MRSA versus SSA [45]	**0.126279**	No
	MRSA versus WOA [37]	0.019059	Yes
	MRSA versus RSA [41]	0.019059	Yes

**Table 12:** Summary of CEC2017 benchmark functions [41].

Type	Number	Function name	*f*_*i*_(*x*^*∗*^)
Unimodal	3	Shifted and rotated Zakharov function	300

Multimodal	4	Shifted and rotated Rosenbrock's function	400
	5	Shifted and rotated Rastrigin's function	500
	6	Shifted and rotated expanded Scaffer's F6 function	600
	7	Shifted and rotated Lunacek bi-Rastrigin function	700
	8	Shifted and rotated noncontinuous Rastrigin's function	800
	9	Shifted and rotated Levy function	900
	10	Shifted and rotated Schwefel's function	1000

Hybrid	11	Hybrid function 1 (*N* = 3)	1100
	12	Hybrid function 2 (*N* = 3)	1200
	13	Hybrid function 3 (*N* = 3)	1300
	14	Hybrid function 4 (*N* = 4)	1400
	15	Hybrid function 5 (*N* = 4)	1500
	16	Hybrid function 6 (*N* = 4)	1600
	17	Hybrid function 6 (*N* = 5)	1700
	18	Hybrid function 6 (*N* = 5)	1800
	19	Hybrid function 6 (*N* = 5)	1900
	20	Hybrid function 6 (*N* = 6)	2000

Composition	21	Composition function 1 (*N* = 3)	2100
	22	Composition function 2 (*N* = 3)	2200
	23	Composition function 3 (*N* = 4)	2300
	24	Composition function 4 (*N* = 4)	2400
	25	Composition function 5 (*N* = 5)	2500
	26	Composition function 6 (*N* = 5)	2600
	27	Composition function 7 (*N* = 6)	2700
	28	Composition function 8 (*N* = 6)	2800
	29	Composition function 9 (*N* = 3)	2900
	30	Composition function 10 (*N* = 3)	3000

**Table 13:** Parameters setting.

Algorithm	Parameters setting
BOA [38]	*a*=0.1, *c*=0.01, *p*=0.6
HHO [42]	*β*=1.5, *E*_0_ ∈ [−1,1]
AOA [47]	*Mop*_max_=1, *Mop*_min_=0.2, *C*=1, *a*=5, *Mu*=0.499
SSA [45]	*c*_1_=rand, *c*_2_=rand
PFA [48]	*u*_1_=−1+2rand, *u*_2_=−1+2rand
TDO [46]	∼

**Table 14:** Statistical results of seven algorithms in the CEC2017 test.

		BOA [38]	HHO [42]	AOA [47]	SSA [45]	PFA [48]	TDO [46]	MRSA
F3	Mean	3.82*E* + 04	1.68*E* + 03	6.91*E* + 04	8.40*E* + 04	4.66*E* + 04	3.77*E* + 04	3.01*E* − 06
	Std	6.97*E* + 03	7.95*E* + 02	1.15*E* + 04	6.59*E* + 03	1.22*E* + 04	3.65*E* + 03	5.54*E* − 07
	Rank	4	2	6	7	5	3	**1**

F4	Mean	9.33*E* + 03	1.23*E* + 02	7.61*E* + 03	1.44*E* + 03	9.80*E* + 01	4.96*E* + 02	7.24*E* + 01
	Std	1.29*E* + 03	3.33*E* + 01	2.45*E* + 03	1.09*E* + 03	1.77*E* + 01	2.16*E* + 01	2.96*E* + 01
	Rank	7	3	6	5	2	4	**1**

F5	Mean	3.49*E* + 02	2.05*E* + 02	2.95*E* + 02	3.50*E* + 02	1.14*E* + 02	6.19*E* + 02	8.24*E* + 01
	Std	2.16*E* + 01	3.62*E* + 01	3.20*E* + 01	4.40*E* + 01	3.11*E* + 01	1.56*E* + 01	2.43*E* + 01
	Rank	5	3	4	6	2	7	**1**

F6	Mean	6.63*E* + 01	5.62*E* + 01	6.21*E* + 01	8.06*E* + 01	1.47*E* + 01	6.00*E* + 02	2.03*E* + 01
	Std	5.76*E* + 00	5.92*E* + 00	6.71*E* + 00	8.84*E* + 00	4.99*E* + 00	3.05*E* − 02	5.92*E* + 00
	Rank	5	3	4	6	**1**	7	2

F7	Mean	5.57*E* + 02	4.98*E* + 02	6.00*E* + 02	7.12*E* + 02	1.34*E* + 02	8.49*E* + 02	1.46*E* + 02
	Std	3.17*E* + 01	6.57*E* + 01	5.66*E* + 01	6.85*E* + 01	3.12*E* + 01	1.47*E* + 01	3.38*E* + 01
	Rank	4	3	5	6	**1**	7	2

F8	Mean	2.93*E* + 02	1.40*E* + 02	2.25*E* + 02	2.72*E* + 02	9.97*E* + 01	9.22*E* + 02	7.56*E* + 01
	Std	1.54*E* + 01	2.13*E* + 01	2.67*E* + 01	4.31*E* + 01	2.66*E* + 01	1.58*E* + 01	2.31*E* + 01
	Rank	6	3	4	5	2	7	**1**

F9	Mean	6.82*E* + 03	4.69*E* + 03	4.50*E* + 03	9.35*E* + 03	2.28*E* + 02	9.01*E* + 02	4.00*E* + 02
	Std	8.69*E* + 02	8.28*E* + 02	7.24*E* + 02	1.85*E* + 03	1.83*E* + 02	8.01*E* − 01	2.11*E* + 02
	Rank	6	5	4	7	**1**	3	2

F10	Mean	7.33*E* + 03	4.35*E* + 03	5.51*E* + 03	7.05*E* + 03	4.98*E* + 03	5.15*E* + 03	3.90*E* + 03
	Std	2.85*E* + 02	7.25*E* + 02	5.83*E* + 02	7.45*E* + 02	9.01*E* + 02	3.62*E* + 02	6.06*E* + 02
	Rank	7	2	5	6	3	4	**1**

F11	Mean	2.19*E* + 03	1.61*E* + 02	1.72*E* + 03	3.91*E* + 03	1.91*E* + 02	1.17*E* + 03	5.60*E* + 01
	Std	6.72*E* + 02	4.86*E* + 01	9.74*E* + 02	1.64*E* + 03	5.28*E* + 01	2.47*E* + 01	2.69*E* + 01
	Rank	6	2	5	7	3	4	**1**

F12	Mean	2.08*E* + 09	7.61*E* + 06	6.27*E* + 09	4.69*E* + 08	1.88*E* + 06	1.85*E* + 05	8.83*E* + 02
	Std	7.43*E* + 08	4.21*E* + 06	2.56*E* + 09	3.76*E* + 08	1.97*E* + 06	9.78*E* + 04	7.27*E* + 02
	Rank	6	4	7	5	3	2	**1**

F13	Mean	3.15*E* + 08	1.51*E* + 05	3.80*E* + 04	8.55*E* + 07	7.54*E* + 04	1.21*E* + 04	2.24*E* + 02
	Std	2.10*E* + 08	9.05*E* + 04	1.71*E* + 04	4.66*E* + 08	4.12*E* + 04	5.52*E* + 03	1.60*E* + 02
	Rank	7	5	3	6	4	2	**1**

F14	Mean	1.19*E* + 05	3.82*E* + 04	5.72*E* + 04	1.50*E* + 06	3.00*E* + 04	2.97*E* + 03	4.32*E* + 01
	Std	7.62*E* + 04	4.25*E* + 04	4.92*E* + 04	1.21*E* + 06	2.94*E* + 04	6.93*E* + 02	1.13*E* + 01
	Rank	6	4	5	7	3	2	**1**

F15	Mean	1.82*E* + 06	6.86*E* + 04	2.35*E* + 04	1.83*E* + 07	3.35*E* + 04	2.40*E* + 03	2.98*E* + 01
	Std	1.46*E* + 06	4.86*E* + 04	1.22*E* + 04	2.37*E* + 07	1.77*E* + 04	5.08*E* + 02	1.67*E* + 01
	Rank	6	5	3	7	4	2	**1**

F16	Mean	3.18*E* + 03	1.55*E* + 03	1.98*E* + 03	2.74*E* + 03	1.00*E* + 03	2.40*E* + 03	1.07*E* + 03
	Std	4.12*E* + 02	3.56*E* + 02	5.09*E* + 02	5.38*E* + 02	2.63*E* + 02	1.34*E* + 02	3.20*E* + 02
	Rank	7	3	4	6	**1**	5	2

F17	Mean	1.22*E* + 03	7.48*E* + 02	9.12*E* + 02	1.20*E* + 03	3.77*E* + 02	1.88*E* + 03	4.41*E* + 02
	Std	2.49*E* + 02	2.19*E* + 02	2.67*E* + 02	3.85*E* + 02	1.71*E* + 02	3.61*E* + 01	2.10*E* + 02
	Rank	6	3	4	5	**1**	7	2

F18	Mean	9.60*E* + 05	6.90*E* + 05	1.29*E* + 06	1.51*E* + 07	2.75*E* + 05	6.11*E* + 04	3.11*E* + 01
	Std	6.22*E* + 05	8.77*E* + 05	1.60*E* + 06	1.51*E* + 07	2.82*E* + 05	2.10*E* + 04	5.54*E* + 00
	Rank	5	4	6	7	3	2	**1**

F19	Mean	4.61*E* + 06	1.46*E* + 05	1.08*E* + 06	4.23*E* + 07	4.45*E* + 04	5.14*E* + 03	2.29*E* + 01
	Std	4.06*E* + 06	1.42*E* + 05	1.39*E* + 05	1.23*E* + 08	3.91*E* + 04	9.69*E* + 02	5.65*E* + 00
	Rank	6	4	5	7	3	2	**1**

F20	Mean	7.29*E* + 02	6.71*E* + 02	6.94*E* + 02	8.59*E* + 02	4.61*E* + 02	2.29*E* + 03	5.30*E* + 02
	Std	9.88*E* + 01	2.01*E* + 02	1.54*E* + 02	2.42*E* + 02	1.52*E* + 02	4.33*E* + 01	1.62*E* + 02
	Rank	5	3	4	6	**1**	7	2

F21	Mean	1.97*E* + 02	4.06*E* + 02	4.87*E* + 02	5.06*E* + 02	2.90*E* + 02	2.41*E* + 03	2.83*E* + 02
	Std	3.01*E* + 01	3.51*E* + 01	5.23*E* + 01	5.36*E* + 01	2.62*E* + 01	9.32*E* + 00	2.52*E* + 01
	Rank	**1**	4	5	6	3	7	2

F22	Mean	4.71*E* + 02	2.39*E* + 03	5.13*E* + 03	4.18*E* + 03	2.08*E* + 02	2.30*E* + 03	1.02*E* + 02
	Std	7.76*E* + 01	2.37*E* + 03	1.21*E* + 03	1.88*E* + 03	7.61*E* + 02	8.09*E* + 00	2.05*E* + 00
	Rank	3	5	7	6	2	4	**1**

F23	Mean	6.97*E* + 02	7.05*E* + 02	9.68*E* + 02	8.60*E* + 02	4.85*E* + 02	2.72*E* + 03	5.11*E* + 02
	Std	5.59*E* + 01	7.35*E* + 01	9.10*E* + 01	1.00*E* + 02	4.09*E* + 01	1.33*E* + 01	4.21*E* + 01
	Rank	3	4	6	5	**1**	7	2

F24	Mean	1.10*E* + 03	8.26*E* + 02	1.14*E* + 03	8.99*E* + 02	5.24*E* + 02	2.88*E* + 03	5.83*E* + 02
	Std	1.68*E* + 02	7.42*E* + 01	1.09*E* + 02	1.37*E* + 02	3.72*E* + 01	1.03*E* + 01	5.29*E* + 01
	Rank	5	3	6	4	**1**	7	2

F25	Mean	1.75*E* + 03	4.11*E* + 02	1.67*E* + 03	7.84*E* + 02	3.97*E* + 02	2.89*E* + 03	3.93*E* + 02
	Std	2.01*E* + 02	1.87*E* + 01	4.55*E* + 02	1.30*E* + 02	1.72*E* + 01	1.09*E* + 01	1.35*E* + 01
	Rank	6	3	5	4	2	7	**1**

F26	Mean	5.21*E* + 03	3.94*E* + 03	6.40*E* + 03	6.30*E* + 03	2.12*E* + 03	3.07*E* + 03	2.38*E* + 03
	Std	1.49*E* + 03	1.10*E* + 03	7.22*E* + 02	1.11*E* + 03	7.10*E* + 02	4.75*E* + 02	4.59*E* + 02
	Rank	5	4	7	6	**1**	3	2

F27	Mean	8.14*E* + 02	6.05*E* + 02	1.34*E* + 03	9.56*E* + 02	5.46*E* + 02	3.21*E* + 03	5.98*E* + 02
	Std	9.81*E* + 01	4.00*E* + 01	2.14*E* + 02	1.65*E* + 02	2.85*E* + 01	6.74*E* + 00	3.98*E* + 01
	Rank	4	3	6	5	**1**	7	2

F28	Mean	3.28*E* + 03	4.62*E* + 02	2.95*E* + 03	1.06*E* + 03	4.31*E* + 02	3.23*E* + 03	4.09*E* + 02
	Std	3.99*E* + 02	2.60*E* + 01	6.15*E* + 02	3.22*E* + 02	1.90*E* + 01	2.10*E* + 01	3.06*E* + 01
	Rank	7	3	5	4	2	6	**1**

F29	Mean	3.04*E* + 03	1.32*E* + 03	2.43*E* + 03	2.64*E* + 03	1.03*E* + 03	3.67*E* + 03	9.64*E* + 02
	Std	4.72*E* + 02	2.56*E* + 02	5.22*E* + 02	6.35*E* + 02	2.35*E* + 02	6.51*E* + 01	2.18*E* + 02
	Rank	6	3	4	5	2	7	**1**

F30	Mean	3.98*E* + 07	1.01*E* + 06	1.47*E* + 07	4.85*E* + 07	4.09*E* + 05	6.59*E* + 03	2.14*E* + 03
	Std	2.31*E* + 07	6.08*E* + 05	1.01*E* + 07	3.75*E* + 07	4.56*E* + 05	3.95*E* + 02	1.05*E* + 02
	Rank	6	4	5	7	3	2	**1**

**Table 15:** The Friedman test results for different algorithms.

Algorithm	Ranking
MRSA	**1.3929**
PFA [48]	2.2143
HHO [42]	3.5714
TDO [46]	5.2857
AOA [47]	5.6429
BOA [38]	6
SSA [45]	6.6071

**Table 16:** The Wilcoxon signed-rank test results for different algorithms.

Comparison	*p* value	*α* = 0.05
MRSA versus BOA [38]	0.000004	YES
MRSA versus HHO [42]	0.000004	YES
MRSA versus AOA [47]	0.000004	YES
MRSA versus SSA [45]	0.000004	YES
MRSA versus PFA [48]	0.039321	YES
MRSA versus TDO [46]	0.000004	YES

**Table 17:** Robot root planning results.

Index	MRSA	RSA [41]	HHO [42]	EO [43]
Best	12.7279	15.5563	12.7279	15.5563
Mean	**14.4250**	16.4049	15.2735	17.8191
Worst	15.5563	21.2132	18.3848	21.2132
Std	1.4606	1.9090	1.6055	2.2311

## Data Availability

The data used to support the findings of this study are available from the corresponding author upon request.
